# Research on Medical Knowledge Graph for Stroke

**DOI:** 10.1155/2021/5531327

**Published:** 2021-03-24

**Authors:** Binjie Cheng, Jin Zhang, Hong Liu, Meiling Cai, Ying Wang

**Affiliations:** ^1^College of Information Science and Engineering, Hunan Normal University, Changsha 410081, China; ^2^School of Humanities and Management, Hunan University of Chinese Medicine, Changsha 410208, China

## Abstract

Knowledge graph can effectively analyze and construct the essential characteristics of data. At present, scholars have proposed many knowledge graph models from different perspectives, especially in the medical field, but there are still relatively few studies on stroke diseases using medical knowledge graphs. Therefore, this paper will build a medical knowledge graph model for stroke. Firstly, a stroke disease dictionary and an ontology database are built through the international standard medical term sets and semiautomatic extraction-based crowdsourcing website data. Secondly, the external data are linked to the nodes of the existing knowledge graph via the entity similarity measures and the knowledge representation is performed by the knowledge graph embedded model. Thirdly, the structure of the established knowledge graph is modified continuously through iterative updating. Finally, in the experimental part, the proposed stroke medical knowledge graph is applied to the real stroke data and the performance of the proposed knowledge graph approach on the series of Trans *∗* models is compared.

## 1. Introduction

With the acceleration of urbanization and social aging, stroke has become one of the diseases with a high rate of death and disability in our country. Stroke is an acute cerebrovascular disease that causes brain tissue loss due to blockage or sudden rupture of blood vessels in the brain. It has the characteristics of high morbidity, mortality, disability, and recurrence. The human brain has an extremely complex nervous system and blood vessels, which brings great challenges to the treatment of brain diseases. So far, the current treatment methods for stroke are still limited and mainly prevent stroke to reduce the occurrence of the apoplexy. Considering that stroke involves many kinds of disease complications, the relationship between medical entities about stroke is complicated. It is impossible to directly use traditional technological means to effectively analyze the medical entity relationship of stroke, which brings a lot of inconvenience to the further prevention and treatment of stroke.

Thanks to the continuous development of Internet technology, the storage and sharing of knowledge has become more convenient. The knowledge of medical field can be integrated and developed through the Internet. More and more science and technology are used in the medical field to contribute to the smart medical field. Knowledge graph is a structured method to express knowledge through visual graphs, which can effectively show some directed lines with mark to depict the association between knowledge. Knowledge graph is essentially a semantic network that reveals the relationship between entities. The nodes in the network represent entities, and the edges between nodes represent the relationship between entities [1]. Knowledge graphs currently have more research and applications in related fields such as in-depth reading, finance, data analysis, medical fields, and other relevant fields. Especially in the medical field, it has very broad application prospects. We can apply the knowledge graph to intelligent question answering, disease-assisted diagnosis, risk assessment, and decision-making systems in the medical field and perform information screening and representation on the information of medical entities thereby establishing a database of medical knowledge relations. Through intuitive relationship expression, the problems in medical diseases can be analyzed more visually, and technical support can be provided for better treatment of diseases. The medical knowledge graph contains a large number of disease knowledge and symptom characteristics, with a wider coverage of entities and concepts and more diverse semantic relationships, which can be used as the basis of machine language cognition. At present, the general medical knowledge graph has more in-depth research and practical application, but there is little attention paid to the knowledge graph for stroke.

According to the China Stroke Prevention and Treatment Report 2019 [2], the current form of stroke disease has become more and more serious, and it is urgent for scientific researchers to brainstorm and contribute to the study of stroke. Therefore, it is very necessary to design a reasonable medical knowledge graph model for stroke, to dig the physical associations related to stroke, and provide a powerful strategy for effective prevention and treatment of stroke further. This paper uses the public information database of the vertical medical website to extract the entities, select the ones with higher confidence to join the knowledge base, and build the connection between the entities. Then, a preliminary medical knowledge graph of stroke is designed through the bottom-up and top-down construction methods. Finally, the structure of the established knowledge graph is modified continuously through iterative updating. A stroke medical knowledge graph with comprehensive coverage, complete structure, and accurate knowledge description is constructed, which lays the foundation for the follow-up stroke intelligent question answering system and auxiliary decision-making system.

The rest of this paper is structured as follows. Some related works are reviewed in Section 2. In Section 3, we design a medical knowledge graph for stroke via knowledge fusion and knowledge graph embedding. In Section 4, we use a real stroke data to verify the performance of the proposed model. Finally, we make a conclusion and give the prospect of future research in Section 5.

## 2. Related Work

From the Semantic Web in the 1990s to the official introduction of the Knowledge Graph in 2012 by Google, the current public knowledge base and a large number of general knowledge graphs have emerged, proving that the research and application of knowledge graphs in various industries and fields have attracted great attention. Knowledge graphs can be simply divided into general knowledge graphs and domain knowledge graphs. There are many general knowledge graphs, large public knowledge bases in the research field, such as DBpedia [3] based on the structured knowledge extracted from Wikipedia entries, connection database YAGO [4] that integrates some Chinese information, and contributions from community partners large-scale cooperative knowledge base called Freebase [5], and Chinese open knowledge graph library OpenKG. Knowledge graph [6] is used by Google in the engineering field on the Google search engine, knowledge graph is used by Baidu for Baidu Search “*Zhixin*,” and *Sogou's* “Knowledge Cube” is used in *Sougo Search*. The medical knowledge graphs studied in this article belong to a category of domain knowledge graphs. Many such knowledge graphs have also been constructed, such as Watson Health of IBM, which mainly uses knowledge graph reasoning and AI analysis of tumor medical images to assist decision-making [3]. And the Chinese medical knowledge graph is also promoted by many domestic institutions such as the knowledge graph constructed by Shanghai Shuguang Hospital mainly used for TCM knowledge QA system and medication recommendations [7] and the Chinese symptom database constructed by East China University of Science and Technology, which has been published on OpenKG [8]. In terms of the construction method of the knowledge graph, a knowledge-based syndrome reasoning method in computer-assisted diagnosis uses the reinforcement learning algorithm to mine the hidden relationship among the entities and obtain the reasoning path. [9] And an improved method for web text affective cognition computing based on knowledge graph constitutes a binary relationship knowledge base. [10] Although the current domestic research on knowledge graphs has gradually improved, various tasks still require a lot of manual intervention to improve, and the research on knowledge graphs in the medical field in our country is still in its infancy.

As mentioned in the China Stroke Prevention and Treatment Report 2019, stroke has become the first year of life lost in China. In 2018, more than 20% of Chinese residents died of cerebrovascular diseases, and the mortality rate has been increasing year by year. The current research on stroke is mainly focused on prevention and treatment [11], so this research uses stroke and related knowledge as the entry point to study the knowledge graph of stroke and construct a medical knowledge graph for stroke.

## 3. Construction of the Medical Knowledge Graph of Stroke

### 3.1. Stroke Medical Knowledge Modeling

The construction of the medical knowledge graph can be divided into two stages. The first is the artificial participation in the construction of the stroke disease dictionary. This part belongs to the description system design. We have investigated the authoritative standard medical term sets at home and abroad, such as the ICD-10 code [12]. According to the medical terminology, we labeled and analyzed the cases and designed the relationship classification system. After comparative evaluation, a stroke disease dictionary was initially constructed. The second stage is the construction of the knowledge graph. Under the guidance of the stroke disease dictionary, the stroke disease-related symptoms, treatment methods, drugs and other attributes, and relationship data are obtained from vertical medical websites and public information databases such as Baidu Encyclopedia. The extracted structured data are manually annotated and automatically extracted to construct the stroke medical knowledge graph ontology. After the knowledge graph modeling and knowledge processing, the semiautomatic construction of the stroke medical knowledge graph is realized.

After determining the construction method, the overall construction framework is formed as shown in Figure 1. The semiautomated construction of the design pattern adopts the cyclic iteration style. Each iteration includes the steps of graph pattern design, knowledge extraction, knowledge graph modeling, and knowledge processing. Such a design can realize the sustainable update of the knowledge graph, so each iteration will produce a new version of the knowledge graph.

### 3.2. Knowledge Graph Pattern Design

To construct a stroke-oriented medical knowledge graph, it is necessary to consider its actual application needs. The stroke medical knowledge graph is mainly used to provide patients with stroke disease self-examination and also provide doctors' medical knowledge base as a reference. The data in the graph contain data on stroke diseases, as well as related treatment methods, symptoms, inspection methods, and drugs in accordance with the requirements of the designated ontology library for manual participation.

Based on medical thesaurus, ICD-10 coding, and other medical terms as entities in the entity resource database, we manually participate in marking stroke diseases and classify them according to different types, respectively, from etiology, diagnostic methods, differentiation, epidemiology, and complications. Past medical history, prevention and recurrence, and other dimensions describe stroke. According to the above methods, a stroke disease dictionary was designed, combined with vertical medical websites, Baidu Encyclopedia, and medical literature to develop a stroke ontology database. In the stroke knowledge graph, the rules in the ontology database are used to constrain the model layer data. The stroke ontology describes all the concepts in the field of stroke and the relationships between them, such as proximity relationships, attribute relationships, and constraints.

There are three methods for constructing the ontology database of the knowledge graph [13]. The first is artificial construction, which is to invite medical experts to participate in the annotation process of the knowledge graph ontology and play a leading role in the description system of the knowledge graph. The second method is automatic construction, which relies on data-driven; the third is semiautomatic construction, which combines manual annotation and data-driven. Taking into account the small scale of the ontology library of stroke medicine implementation graphs, the third method can obtain the ontology with higher quality and save human resources. This article uses the third method to construct the ontology library. First, use manual intervention to build a simple stroke ontology database for the stroke disease dictionary, then extract pattern data with guaranteed accuracy from the knowledge processing process in the subsequent steps, and add it to the stroke ontology database after manual verification is correct.

According to this construction process, after extracting high-confidence data from the vertical medical website and Baidu Encyclopedia, the entities, relationships, and attributes covered by the ontology library are refined, and the value range of each attribute is finally clarified.  Figure 2 shows the information of the disease entity category.

### 3.3. Data Source

In the process of constructing a stroke medical knowledge graph, a key step is knowledge extraction, and data confidence is the basis for whether knowledge extraction is efficient and accurate.  Figure 3 shows the knowledge extraction process of the stroke medical knowledge graph.

Currently, there is a lack of a stroke medical knowledge graph in the public knowledge base, so the data sources for constructing a stroke knowledge graph in this article mainly include vertical medical websites, crowdsourced encyclopedia websites, and general knowledge graphs in the public knowledge base.

Two medical websites were selected in this study: Xunyiwenyao.com, which is a doctor-patient communication platform. Doctors and hospitals participate voluntarily. The content contained in the website is highly professional and accurate. The degree is high, mainly including basic medical information data, health information, and medical questions and answers; *Dingxiangyuan* is a data service platform that includes disease encyclopedias, medication specifications, and medical science popularization. This study combined the open source data of these two vertical medical websites as the main source of the data layer of the stroke knowledge graph.

Baidu Encyclopedia is the largest crowdsourcing website in China. It is basically crowdsourced by experts in various fields. The structured data contained in it are the best supplement to the knowledge graph data layer. Baidu Encyclopedia is aimed at medical entity entries. The explanatory text contains a lot of information such as disease nicknames and context, and this part of the data has high value.

The public knowledge base, the Chinese symptom database of East China University of Science and Technology from *OpenKG* used in this article, extracts stroke nodes and relationships from it. This part can also complement the ontology database and data layer of the knowledge graph.

Different data sources require different processing methods. Since the data on vertical medical websites and crowdsourcing websites are structured, this article uses distributed crawlers to automatically crawl medical data. The knowledge graph from the public knowledge base can be directly integrated. After obtaining the data from the three sources, it is saved as a lightweight JSON file. For this kind of data, the first task is to clean up the data and clean up the default, garbled, and illegal characters.

### 3.4. Knowledge Fusion

The knowledge fusion in the knowledge graph can be realized in many ways. This study uses the two perspectives of entity attribute alignment and entity linking with the help of the similarity calculation method to carry out the knowledge fusion of the stroke knowledge graph. Entity alignment refers to merging the entities in the knowledge base of heterogeneous data sources into an entity with a globally unique identifier in the real world [14] and then linking the aligned entities to the stroke knowledge graph. Since this paper proposes to formulate a stroke disease dictionary, the entity alignment step has been completed in the data extraction stage, so the entity attribute alignment stage is mainly to align the attributes.

#### 3.4.1. Attribute Alignment

The effect of this step of attribute alignment is to improve the accuracy of entity links. Since there are few attributes in the stroke field, this paper constructs an attribute mapping table based on the constraints of the stroke ontology library and aligns the different expressions of the same attributes of the same entities.  Table 1 shows some attribute alignment mappings of heterogeneous data sources.

After the attributes of heterogeneous data sources are aligned, the attribute values are standardized according to the constraint specifications in the model layer. This research divides the attributes as follows: numeric type, numeric interval type, entity object list type, string type, and Boolean type. These attribute values are standardized and structured according to the following constraint specifications:

- The unit of measurement for numeric attribute values is unified
- Space characters and line breaks in the attribute value of string type must be deleted
- For interval attribute values, keep the upper and lower limits and store them in the list
- The attribute values of the entity object type are all stored in the list, and no attribute alignment operation is performed

#### 3.4.2. Entity Linking

After completing the work of attribute alignment and normalizing attribute values, choose to calculate the semantic similarity of the result after attribute alignment to determine the relationship with the entity nodes in the knowledge graph and then decide whether to link to the knowledge graph. In stroke medical entities, this study calculates the similarity of the abovementioned different types of attribute values to determine whether to link to the entities in the knowledge graph. For two entities *W1* and *W2*, the corresponding aliases and names merged into the name set are *S1* and *S2*, respectively. Calculate the similarity according to the following equation and links with high similarity to entities in the knowledge graph:

(1) $$\begin{array}{c} \text{Sim}\left(W_{1},W_{2}\right)=\frac{k}{1+N}\max\left(\sum_{i\in W1}^{N}\sum_{j\in W2}^{N}\frac{2\times lcs\left(i,j\right)}{L_{i}+L_{j}}\right). \end{array}$$

Among them, *lcs*(*i*, *j*) represents the length of the largest common subsequence of the names *i* and *j*, N is an adjustable parameter, *L*_*i*_ and *L*_*j*_ represent the length of the word in *W*_*1*_ and *W*_*2*_ in the entity, and *k* is a weight parameter to avoid the influence caused by the high similarity of the name set.

#### 3.4.3. Knowledge Merger

Knowledge merging in the medical knowledge graph is to integrate structured knowledge and knowledge in the public knowledge base into the existing knowledge graph. The aforementioned Chinese symptom database is such a source of knowledge that can be incorporated into the stroke knowledge graph. The knowledge it possesses conforms to the knowledge norms and has high practicality and high knowledge quality.

This article will refer to the method of knowledge merging for LOD by Mendes et al. [15] and conclude that the process of merging the public knowledge base into the stroke knowledge graph is knowledge extraction, concept matching, entity alignment, and knowledge evaluation. The two steps of concept matching and entity alignment are to normalize the knowledge extracted from the Chinese symptom database with the artificial stroke disease dictionary, and the knowledge evaluation is used to detect the consistency and accuracy of the extracted knowledge.

### 3.5. Knowledge Graph Embedding

In the medical knowledge graph, each piece of medical knowledge can be represented by a triple such as 〈head, relation, tail〉, where head represents the head entity node, tail represents the tail entity node, and relation represents the relationship between nodes. For example, the results of the triple representation of ischemic stroke are shown in Table 2. At the same time, all the triples in Table 2 are combined to obtain a partial knowledge graph of “ischemic stroke,” as shown in Figure 4. The knowledge graph modeling is to graph the relationship between the head and tail entity nodes and the entities to a continuous low-dimensional vector space and represent them as entity vectors, so that the semantic structure information between the triples can be saved and used to calculate the similarity between entities. This article uses TransE [16] and TransD [17] models that are currently widely used in knowledge representation. The TransE model is the first model proposed by the Trans series, which mainly associates entity nodes by mapping the word vector to a low-dimensional space to calculate the similarity. The TransD model is a more advanced generalization of the TransE model. The latter is a special case of the former. Therefore, this paper will verify which model is better for the proposed knowledge graph construction.

The TransE model is the most representative translation model. For the given triples, the relation is interpreted as the translation vector from head to tail; when the triple of 〈head,relation, tail〉 is established, the relationship between nodes is shown like head+tail»relation. Otherwise, the tail node should not be linked to the other end of the head entity node and the relationship. The specific function formula is shown in the following equation:

(2) $$\begin{array}{c} f_{r}\left(h,t\right)={\left\|h+r-t\right\|}_{L_{1}/L_{2}}. \end{array}$$

Among them, *L*_1_/*L*_2_ refers to the distance of *L*_1_ or *L*_2_ when calculating. *L*_*1*_ represents the translation distance from the *r* vector to the *h* vector. *L*_*2*_ represents the translation distance from the *r* vector to the *t* vector. Due to the few model parameters and low computational complexity, the TransE model can handle one-to-one relationships well, but its performance is insufficient when dealing with one-to-many or even many-to-many relationships. Therefore, this article will also combine the TransD model and the TransR model that has been extended to TransE to perform knowledge representation processing on the triples of the subdivided medical knowledge graph.

The TransD model believes that the head and tail entity nodes in the triplet represent different semantics after the connection relationship. Therefore, the model uses the mapping matrices *M*_*h*_ and *M*_*t*_ to graph the head and tail entities to the relationship space and decomposes the mapping matrix of each relationship into the product of two vectors, and the function formula is shown in the following equation:

(3) $$\begin{array}{c} f_{r}\left(h,t\right)={\left\|M_{h}h=r-M_{t}t\right\|}_{L_{1}/L_{2}}, \end{array}$$

where *M*_*h*_=*r*_*p*_*h*_*p*_+*I*, *M*_*t*_=*r*_*p*_*t*_*p*_+*I*, and *I* is the identity matrix. Obviously, we can see that *M*_*h*_ and *M*_*t*_ are related to entities and relationships. The calculation speed of the model can be improved through vector operation conversion.

### 3.6. Knowledge Processing

#### 3.6.1. Medical Ontology Model Layer Inspection

In the case that the new version of the ontology model layer formed by iteration and the existing model layer exists at the same time, the type and value constraints of the data that have been fused into the graph are applied to make the data layer meet the ontology model specifications defined in the layer. This article generates a rule database based on the model layer constructed by the stroke disease dictionary to test the data layer. The rule base includes entity type detection and attribute value interval detection.

#### 3.6.2. Graph Update

In Section 3.2, this article developed a stroke disease dictionary based on actual needs and defined the model layer of the stroke knowledge graph based on the dictionary. However, it is difficult to ensure that the model layer can cover all data patterns in practical applications. Among the data obtained from heterogeneous data sources, there are some data patterns that are not clearly defined but have research value. We will generalize new data patterns from these new data and improve and supplement the stroke ontology database previously constructed.

Since the stroke medical knowledge graph constructed in this paper is different from the general medical knowledge graph, we have manually intervened the boundaries of the knowledge graph to ensure that the knowledge graph will not extend infinitely in breadth. For the relationship types that already exist in the current model layer and the head and tail node types are also known, they are linked to the existing entity relationships in the stroke knowledge graph through the semantic similarity calculation in Section 3.4. If there is no corresponding entity relationship, add a new entity relationship directly in the pattern layer; another case is that only one of the connected head and tail entities can find the corresponding relationship type in the pattern layer. This unknown type will appear in this article, the entity is extracted, the number of occurrences is calculated, and then its entropy value is normalized. The relationship type with larger entropy value and the entity type is added to the model layer as a candidate model. The stroke knowledge graph constructed by this loop iteration method will be relatively stable and complete, and the subsequent update direction depends on the application requirements. The follow-up knowledge graph update work can use deep learning models to learn the cascaded R–CNN and a correlation filter learning model of real data [18,19].

#### 3.6.3. Quality Evaluation

The quality evaluation of the knowledge graph mainly quantifies the confidence of the knowledge in the graph and discards the knowledge with low confidence to ensure the quality of the entire knowledge graph [20]. In this paper, a semiautomated hierarchical ontology metric based on semiotics combined with manual calculation is used to evaluate the constructed stroke medical knowledge graph.

## 4. Experiment

### 4.1. Dataset

The experimental data in this article consist of two parts. One part of the data comes from the stroke-related description text data crawled from Xunyiwenyao.com and Baidu Encyclopedia by writing a crawler program; the other part is public Chinese obtained from OpenKG a triad of partial knowledge about stroke which is extracted from the symptom database and obtained a total of 4113 related entities related to stroke, with 8 attribute types (name of disease, introduction, susceptible population, etiology, treatment, treatment cycle, preventive measures, and cure probability) and 10 types of entity relationship. Specific information is as follows.  Table 3 shows that there are 7 types of entities, and the specific type information is shown in Table 4.

### 4.2. Experiment Analysis

In this paper, the construction of the stroke knowledge graph is firstly through the semiautomatic labeling method plus human participation and the development of a stroke disease dictionary, combined with international general medical terminology and other professional information to construct a preliminary model layer. Then, a crawler is designed, combined with data cleaning to screen and crawl the open text data of *Xunyiwenyao.com*, *Dingxiangyuan.com*, and *Baidu Encyclopedia*, and the knowledge is extracted from the Chinese symptom database constructed by East China University of Science and Technology as stroke medicine. To supplement the knowledge graph, store these knowledge triples in the Neo4 J graph database. By means of knowledge fusion, knowledge graph embedding, and knowledge processing, iteratively update the stroke knowledge graph so that it is continuously improved while retaining the boundaries, forming the domain closure of the stroke knowledge graph.

Figure 5 is a partial knowledge graph of stroke disease information. The constructed stroke medical knowledge graph belongs to the Chinese knowledge graph, so the content shown in Figure 5 is Chinese. For example, hypertensive patients belong to the high-risk population of stroke diseases. In the database, you can query the information on the antihypertensive drugs of the predisposing factors of stroke and high blood pressure in the database. The database will return as follows.  Figure 6 shows the subgraph. Since the *Xunyiwenyao* website and the *Dingxiangyuan* website belong to a doctor-patient communication platform, there will be consultations from most patients to medical experts. This part of the data is also crawled down in this study, and an intelligent question-and-answer system can be initially constructed.

### 4.3. Comparative Analysis of Trans Series Models

This paper selects the TransE model and the TransD model to express the knowledge of the knowledge graph. The experiment will select the TransD model as the main research model to compare with the TransE model and use the two models, respectively, to randomly extract the 200-dimensional head and tail entities and relationships from the knowledge graph. The triple vector is used for training. The experimental verification method is cross-validation, using 70% of the randomly selected vectors as the training set and 30% of the data as the test set. The three values of precision, recall, and F1 are used as evaluation indexes; these three indicators are mainly used to evaluate the effects of these two models in this article, so as to choose which model to use. The experiment was repeated 10 times, and the average value was taken as the final model evaluation result.

The experimental results are shown in Table 5. It is not difficult to see that the performance of the TransD model is better than that of the TransE model. In terms of accuracy, recall, and F1 value, the TransE model has different degrees of improvement over the TransD model. Therefore, in the medical knowledge graph with complex semantic relationships, the TransD model graphs the head and tail entities to the low-dimensional vector space of the relationship through the mapping matrix to represent the semantic structure and better captures the nonlinearity between structured knowledge. Relationships reduce the loss of the vectorization process of physical nodes. This method is more reasonable and can play a greater role in the stroke ontology database.

## 5. Conclusion

Stroke is a disease that urgently needs to reduce the risk of treatment. The proposed stroke-oriented medical knowledge graph can effectively discover the associations between medical entities and establish a certain foundation for subsequent intelligent question-and-answer and medical assistance decision-making systems. Firstly, according to the actual application requirements, we manually participate in the development of a stroke dictionary using semiautomatic annotation and build a model layer of the knowledge graph combined with international standard medical terminology such as ICD-10. Secondly, the improved entity similarity measure is used to perform knowledge fusion on the processed stroke information and link the relationships between entities to the nodes of knowledge graph. Then, we perform the knowledge representation by the knowledge graph embedded model, and the constructed knowledge representation is updated and iterated at the same time to more accurately express the association between entities. In addition, the constructed knowledge graph of stroke already can be used in general medical question answering systems.

At present, there are a few medical knowledge graphs that have been applied to the actual medical scenarios, and their confidence has always been controversial. It is also a problem that needs to be solved as to how to systematically construct the medical knowledge graph for stroke. In future research work, we will focus on the application-level development of the stroke knowledge graph, such as exploring how to further intelligentize the question answering system and combine the deep learning model to extend the intelligent diagnosis.

## Figures and Tables

**Figure 1:** Stroke medical knowledge graph construction framework diagram.

**Figure 2:** Partial structure of disease ontology.

**Figure 3:** Knowledge extraction flowchart of stroke medical knowledge graph.

**Figure 4:** Example of ischemic stroke knowledge graph.

**Figure 5:** Part of ischemic stroke knowledge graph.

**Figure 6:** Subfigure of high blood lipid entity structure.

**Table 1:** Partial attribute alignment mapping table of heterogeneous data sources.

Sample	Data source	Original attribute	Aligned attributes
1	https://http://www.xywy.com/	Treatment department	Treatment department
	https://www.dxy.cn/	Registration department	
2	https://http://www.xywy.com/	Alias	Nickname
	https://www.dxy.cn/	Nickname	

**Table 2:** Ischemic stroke description triad.

Head	Relation	Tail
Ischemic stroke	Nickname	Cerebral infarction
Ischemic stroke	Susceptible population	People with high blood pressure
Ischemic stroke	Susceptible population	Middle-aged and elderly
Ischemic stroke	Clinical manifestations	Hemiplegia
Ischemic stroke	Clinical manifestations	Hard to swallow
Ischemic stroke	Clinical manifestations	Numbness of the contralateral limb
Ischemic stroke	Clinical manifestations	Sensory disturbance
Ischemic stroke	Clinical manifestations	Aphasia

**Table 3:** Knowledge graph entity relationship type.

Entity relationship type	Example	Number of relationships
Department	<*Stroke, belongs to, Neurology*>	551
Commonly used drugs	*<Ischemia stroke, commonly used drugs, mannitol>*	2035
Suitable to eat	*<lschemic stroke, suitable to eat, rich in plant protein>*	386
Drugs on sale	*<lschemic stroke, medicines on sale, Tongmai granules>*	527
Examination	*<Ischemia stroke, examination, brain MRI examination>*	1029
Avoid eating	*<Ischemia stroke, avoid eating, high greasy fat>*	793
Recommended drugs	*<Ischemic stroke, recommended drugs, Tongmai granules>*	1348
Recommended recipe	*<lschemic stroke, recommended diet, easy to digest>*	410
Symptom	*<Ischemia stroke, symptoms, deflection of tongue extension>*	949
Complication	*<lschemic stroke, complications, pulmonary embolism>*	1202

**Table 4:** Stroke knowledge graph entity type.

Entity type	Example	Number of entities
Diagnostic inspection items	Head CT or brain MRI	301
Treatment department	Internal medicine, neurology	10
Disease	Ischemic stroke, hemorrhagic stroke	798
Medicine	Urokinase	2035
Food	Light and easy to digest food	507
Disease symptoms	Deviated tongue, sticking out	462

**Table 5:** Trans series model parameter table %.

Model	Precision	Recall	F1
TransE	71.7	62.9	67.0
TransD	85.8	85.45	85.6

## Data Availability

The data used to support the findings of this study are included within the article (https://www.xywy.com).
